This article has been retracted.

# Depth Vision-Based Assessment of Bone Marrow Mesenchymal Stem Cell Differentiation Capacity in Patients with Congenital Scoliosis

**DOI:** 10.1155/2022/4890008

**Published:** 2022-04-12

**Authors:** Ning Liang, Qiwen Zhang, Bin He

**Affiliations:** The Third Affiliated Hospital of Zunyi Medical University (Zunyi First People's Hospital), Zunyi, Guizhou 563000, China

## Abstract

Congenital scoliosis (CS) is a lateral curvature of one or more segments of the spine due to spinal dysplasia during fetal life. CS is clinically defined as a curvature of the spine >10° due to structural abnormalities of the vertebrae during the embryonic period. Its etiology is unknown, but recent studies suggest that it may be closely related to genetic factors, environmental factors, and developmental abnormalities. The induction methods and modern applications of bone marrow MSCs provide a reference for in-depth human research on the induction of differentiation of bone marrow MSCs into osteoblasts. In this paper, by reviewing and organizing the literature on bone marrow MSCs, we summarized and analyzed the biological properties and preparation of bone marrow MSCs, the methods of inducing osteoblasts, the applications in tissue engineering bone, the problems faced, and the future research directions and proposed a method to assess the differentiation ability of bone marrow MSCs in patients with congenital scoliosis based on depth visual characteristics and the change of the method. The method reveals and evaluates the multidirectional differentiation potential of bone marrow MSCs, which can be induced to differentiate into osteoblasts in vitro and can be used to construct bone tissue engineering scaffolds in vitro using tissue engineering techniques. Based on the properties of bone marrow MSCs, their application in congenital scoliosis patients for trauma repair, cell replacement therapy, hematopoietic support, and gene therapy is quite promising. It is necessary to carry out research on the mechanism of osteogenic differentiation of bone marrow MSCs to provide guidance and reference value for their induced differentiation into osteoblasts.

## 1. Introduction

Congenital scoliosis (CS) is a three-dimensional deformity of the spine due to the abnormal development of the vertebral structures resulting in a coronal curvature of more than 10°. CS is often combined with rib and thoracic deformities that affect the patient's appearance and lead to irreversible pulmonary impairment [1–3]. In addition, other systemic malformations, including spinal cord, heart, kidney, and gastrointestinal system, can be observed in CS patients. The incidence of combined congenital defects of other systems in CS patients is 40%–66%. The current reports on concomitant malformations in CS are mostly limited to the incidence and classification of intraspinal and cardiac malformations, and the incidence of concomitant malformations reported in studies varies widely. A comprehensive retrospective analysis of the clinical features of CS combined with other systemic malformations was performed to explore the possible intrinsic link between the concomitant malformations of each system. The pathogenesis of CS is related to vertebral body formation, which develops from embryonic somatic segments. Most scholars agree that both genetic and environmental factors that can affect the normal development of the somites are likely to contribute to CS. The extensive and sequential involvement of the somites and subsequent development will result in different types of vertebral abnormalities and corresponding clinical manifestations. The current research focuses on environmental factors: maternal gestation, especially during somite formation, may have an impact on gene signal expression and epigenetics; genetic factors: based on the constancy of the location of specific genes encoded in vertebrates (e.g., vertebral body formation genes), identification of candidate genes by homozygosity of animal and human gene sequences, and population-based single nucleotide polymorphism (SNP). Nucleotide polymorphisms (SNPs) were screened in the population [4–7]. With regard to environmental factors, many physicochemical factors were found to cause vertebral developmental malformations in animals, such as high heat, organophosphorus pesticides, and drugs that can induce vertebral malformations in rodents; NO can induce vertebral developmental malformations in chickens. Risk factors for vertebral malformations in humans have been reported: in a controlled analysis of 228 patients with CS between the ages of 0 and 50 years and 268 individuals with normal spines, risk factors were considered to include maternal insulin-dependent diabetes mellitus, valproic acid, alcohol, smoking, hyperthermia, twin pregnancies, artificially assisted reproductive techniques, and in vitro fertilization.

The rise of assisted reproductive technology has led to an increase in the incidence of multiple pregnancies and an increasing emphasis on epigenetics (i.e., no changes in DNA sequence but changes in gene expression resulting in different phenotypes). The genes involved in the typing of vertebral defects are shown in Figure 1. Because of this technique, methylation of nutrients or histone modifications, for example, can be detected allowing epigenetics to explain the occurrence of congenital malformations and some syndromes. The detection of genetic predisposition divides CS into syndromic and disseminated nonsyndromic types. Most CS tends to be disseminated, except for the typical syndromes, which have a tendency to cluster in families and are considered autosomal recessive by linkage analysis. A review of identical and heterozygous twins who developed CS was summarized through study reports of CS family lines, and it was concluded that disseminated CS tends to be a polygenic genetic disorder influenced by environmental, epigenetic influences. Dissemination leads to a lack of typical family lines making screening for single nucleotide polymorphisms more appropriate for CS studies. Genes associated with vertebral development in mice have been elucidated [8], and with the completion of human exome and whole-genome sequencing, gene-disease association analysis has become a research hotspot, and more progress has been made in association analysis of SNPs at genetic loci for CS. The SNPs loci associated with CS genetic susceptibility are: (1) syndromic type: SCD-associated loci include: DLL3, MESP2, LFNG, HES7, TBX6; STD-associated loci include: MESP2; (2) nonsyndromic type: PAX1 polymorphism is associated with CS genetic susceptibility; WNT3A polymorphism has insufficient evidence to be associated with CS genetic susceptibility. Regarding the loci associated with CS genetic susceptibility in the Chinese Han population, HES7, TBX6, and LMX1A were identified. Although CS has been suggested to be autosomal dominant or recessive, the mode of inheritance is generally unclear, and the current mainstream research supports polygenic inheritance of CS. The genetic pattern of spondylus costal dysostosis (SCD), a rare syndrome associated with CS, is better understood, as SCD can be divided into four subtypes, all of which are autosomal monogenic recessive, with mutations in the DLL3 type. These genes are all related to the NOTCH signaling pathway, which plays an important role in organogenesis, development, and apoptosis during the early development of various tissues and organs. Osteogenesis within the cartilage is significantly restricted [9–11]. The study of SCD, a genetic disease with spinal deformity, provided important information on the genetic pattern of CS, suggesting that these genes play an important role in the normal development of the spine. Through various sequencing tools such as whole-genome sequencing, whole-genome exon sequencing, and whole-genome association analysis, combined with various model animal experiments such as zebrafish model and point mutant mice, researchers have screened some pathogenic genes associated with CS pathogenesis. DLL3 was used as a candidate gene, and sequencing of the DLL3 gene in 46 CS patients identified a new highly conserved missense mutation (S225 N). Validation experiments in a point mutant mouse model revealed that HES7, an effector gene of NOTCH, encodes a HES transcriptional repressor, and when a single dose of HES7 is insufficient, it can cause defects in embryonic somatic segment development by interfering with fibroblast growth factor (FGF) expression and eventually cause CS malformations in mice. The WNT3A gene may also be associated with somite development and CS. The WNT3A/*β*-catenin pathway regulates the expression of somite boundary determination genes MESP2 and Ripply2 by activating the activity of DLL1 and TBX6, and ultimately determines the boundary formation during somite development. By whole-genome exome sequencing and comparative genomic hybridization microarray, the TBX6 gene was targeted for possible association with CS. TBX6 gene, known as T-box6, is located at 16p11. The translation product is involved in mesoderm development as a transcription factor and transcriptionally regulates the morphogenesis process. The discovery of TBX6 could explain the formation of CS in 11% of the cases studied.

Currently, autologous bone graft, allogeneic bone graft, and artificial bone substitute graft are the main treatments for bone defects, but all methods have limitations that lead to poor clinical outcomes. Autologous bone harvesting is limited and more invasive, which can easily lead to postoperative infections and complications. Allogeneic bone grafting, although not a limited source, carries a potential risk of immune response. Therefore, rapid and safe methods for bone defect repair have become a research direction in the field of bone injury in recent years [12]. BMSCs (bone marrow mesenchymal stem cells) originate from mesodermal cells and are multipotent stem cells with multispectral differentiation, high proliferative capacity, and easy gene transfection, which can differentiate into osteoblasts, chondrocytes, adipocytes, and neuronal cells under different conditions. BMSCs are easy to obtain, have low immunogenicity, are easy to transfect, and can effectively suppress immune rejection after allogeneic transplantation by transfecting BMSCs with specific genes. Therefore, BMSCs are important source cells for regenerative medicine and tissue engineering. BMSCs are multipotent stem cells that can differentiate into a variety of tissue cells, have weak immunogenicity, and can be easily transfected with exogenous genes, making them a hot vector cell for tissue engineering research and showing a bright future in the field of gene therapy and cell therapy. As ideal target cells for gene therapy, BMSCs have many biological properties such as high metabolic viability, favorable recombinant protein secretion, multi-directional differentiation potential under different induction conditions, and strong in vitro expansion ability. In order to promote the sustainable transformation of BMSCs into osteoblasts, it is necessary to maintain the continuous action of osteogenic inducers outside [13]. They are currently used extensively for cell and tissue replacement therapy in a variety of diseases. However, with the continuous research on BMSCs, it has been found that the number and proliferation and differentiation potential of BMSCs decreases with age, limiting the wide application of autologous BMSCs for transplantation. Therefore, the search for new sources of MSCs is one of the hot spots of stem cell research at home and abroad in recent years. BMSCs' biological characteristics are derived from bone marrow stroma and have the characteristics of mesenchymal and endothelial cells, capable of expressing a variety of antigens, including adhesion factors, growth factors, many receptors and integrins, but not their specific antigens. MScs play the role of supporting and nourishing hematopoietic cells. BMSCs play a role in supporting and nourishing hematopoietic cells, a primitive cell subpopulation of nonhematopoietic origin with a highly self-replicating, multispectral differentiation potential. BMSCs have a strong proliferative and multi-directional differentiation potential and play an important role in bone metabolism, with a strong osteogenic potential and maintain the ability to repair bone necrosis [14]. BMSCs are ideal seed cells for bone tissue engineering research. Moreover, BMSCs can easily accept exogenous gene introduction and have promising applications in hematopoietic reconstruction, tissue repair, and gene therapy, making them highly promising vector cells for gene therapy. Currently, the commonly used methods for the isolation and purification of BMSCs include whole bone marrow applanation culture and density gradient centrifugation. While BMSCs are identified mainly with the help of their surface antigenicity, BMSCs express a variety of surface proteins such as CD29 and CD44 after cell apposition attachment but do not express hematopoietic stem cell surface markers such as CD14 and CD34. These surface antigens are immunologically specific, with low expression of the major histocompatibility complexes MHC I and MHC II and no expression of major costimulatory molecules such as CD40, CD80, and CD86. Thus, allogeneic transplantation of BMSCs does not cause rejection. Therefore, BMSCs have received increasing attention and become the main seed cells for gene therapy, cell therapy, and tissue-engineering-related research, and have good application prospects [15].

Visual depth feature extraction and disease diagnosis based on biomedical images have become an integral and increasingly important part of healthcare. Magnetic resonance image (MRI), Positron emission tomography (PET), Computer tomography (CT), cone beam CT, 3D ultrasound imaging, and other medical imaging technologies are widely used in clinical examination, diagnosis, treatment, and decision-making. The cell morphology of BMSCs under transmission electron microscopy is shown in Figure 2. In this paper, we propose a visual depth feature-based method to evaluate the differentiation capacity of bone marrow MSCs in patients with congenital scoliosis, which uses artificial intelligence deep learning methods to analyze and process these large-scale medical image data and provides scientific methods and advanced technologies for screening, diagnosis, treatment planning, treatment image guidance, efficacy assessment, and differentiation capacity evaluation of bone marrow MSCs in patients with congenital scoliosis in clinical medicine. It is a major scientific problem and a key technology of cutting-edge medical imaging that needs to be solved in the field of medical image analysis.

## 2. Related Work

### 2.1. Congenital Spinal Deformity

Congenital vertebral deformities are widely recognized by clinical practitioners through the scoliosis deformities they cause. Winter et al. based on radiographic typing is widely accepted and applied by scholars to classify CS into vertebral body formation disorders, vertebral segmentation defects, and mixed types [16, 17]. Combined with genetic typing with the development of genetics, researchers recognized that CS is genetically related, and in order to recognize uniformity, the International Federation of Spinal Deformity and Scoliosis proposed a guided typing system on congenital vertebral defects, which proved to have high reliability and validity. This typing first classifies congenital vertebral defects into single defects, multiple localized defects (<10 affected vertebrae), and multiple extensive defects (≥10 affected vertebrae). Fractionation based on frontal and lateral radiographs can evaluate the vertebral body and the vertebral arch, but it does not show well for the posterior spinal complex and severe and complex scoliosis. With the development of CT and the popularity of 3D CT, 3D fractionation of CS was proposed. The first step: the vertebral defects were determined on the basis of single and multiple occurrences to determine whether the vertebral body was consistent with the posterior relationship; the second step subdivided the location and morphology of the formation of the disorder; the third part looked at whether there was a segmentation disorder, again subdivided according to the location, morphology, and whether the anterior and posterior sides were consistent. Eventually, CS was divided into: (1) single consistent defects (hemivertebrae, cuneiform vertebrae, butterfly vertebrae, etc.); (2) multiple consistent defects (simultaneous appearance of hemivertebrae, cuneiform vertebrae, or butterfly vertebrae in adjacent or different locations); (3) complex inconsistent defects (mismatch complex, mixed complex): this type still needs further in-depth differentiation; (4) subsegmental defects (can be subdivided according to location, direction, and rib relationship subdivision). However, there are no studies related to the etiology, embryology, and the expected progression of 3D subtypes.

Progression of scoliosis tends to occur during peak growth (birth to late 4 years and adolescence), and CS is no exception. The risk of progression is currently considered low for fully blocked vertebrae, cuneiform vertebrae, and unsegmented hemivertebrae; partial or fully segmented, especially multiple hemivertebrae, are more likely to progress; unilateral nonsegmented thoracic segments, especially combined with contralateral hemivertebrae, progress rapidly, and there is a lack of systematic reports on the prognosis of complex mixed forms. After a period of observation and evaluation, the child can also be prepared for surgery accordingly [18]. Conservative treatment is mainly divided into cast and brace correction, and halo ring continuous traction. The second “China-US TSRH Orthopedic Surgeon's Association” has dedicated a series of lectures to halo ring and cast correction: halo ring traction can be equipped with mobile carts, play apparatus, and even special traction beds, with electronic devices that can adjust and monitor the amount of traction force recorded. It is believed that halo ring traction can be used at any age, for any type of scoliosis, and even for patients who have failed after surgery. In addition to contraindications (e.g., intramedullary occupancy and spinal stenosis), subjective intolerance, these limitations include stent height that is too high to pass indoors. Fletcher et al. used a series of casts on 29 patients with IS and CS over 50°, successfully delaying the first surgery by an average of 39 months, avoiding the need for propping of growth rods in 21 children, and in follow-up of 11 children with involvement of multiple segments confirmed the effectiveness of brace treatment. It is important to note that bracing or cast immobilization is not a lateral compression of the thorax; rotational compression is the key, as otherwise cardiopulmonary function and rib development are easily compromised. The biggest benefit of conservative treatment is that it delays the timing of surgery and reduces the number of nonfusion surgeries [19]. For patients who have poor cardiopulmonary function or whose cardiopulmonary function is greatly affected by plaster support fixation, halo ring traction is more recommended; conservative treatment cannot cure the disease, and strict follow-up observation is needed during and after treatment.

### 2.2. Machine Learning Instructional Evaluation

Bone marrow stromal cells are a heterogeneous population of many cells, among which exist mesenchymal stem cells, which are adult stem cells with self-renewal, replication, and multi-directional differentiation potential [20]. Bone marrow MSCs can differentiate in two directions, osteogenesis and lipogenesis, and maintain a dynamic balance between the two. Once the physiological processes of osteogenesis and lipogenesis are disturbed, a number of metabolism-related and developmental disorders will result. In diseases such as osteoporosis and age-related bone loss, the reduction of bone tissue is often accompanied by a significant accumulation of adipose tissue. In some diseases characterized by high bone mass, for example, increased abnormal bone formation and increased ossification are often accompanied by a decrease in intra-tissue fat content. The effects of abnormal differentiation of BMSCs are particularly evident during the growth spurt. Due to significant changes in the amount of osteogenesis in adolescents, abnormal osteogenic differentiation can lead to a variety of clinical disorders, such as osteogenesis imperfecta, osseous malocclusion, and abnormal bone age. In addition, trauma, severe infection, tumor resection, or skeletal abnormalities can cause bone defects, resulting in abnormal bone mass. Therefore, it is important to explore the balance mechanism between osteogenic differentiation and lipogenic differentiation for the elucidation of the pathological mechanism and treatment of bone-related diseases as a clinical guide.

The source of BMSCs is limited, and the content of BMSCs in bone marrow is very small, only 0.01%–0.1%, but BMSCs have strong proliferative ability in vitro, and the number of passages has little effect on the proliferation ability of cells. The morphology of primary and passaged bone marrow MSCs is shown in Figure 3. Currently, the international methods for in vitro isolation and culture of BMSCs mainly include whole bone marrow apposition, density gradient centrifugation, flow cytometry sorting, and immunomagnetic bead method. Among them, the most commonly used methods are whole bone marrow culture and density gradient centrifugation. The flow cytometry sorting method and immunomagnetic bead method use fluorescence and magnetic beads to label the surface antigens of BMSCs, which have the advantages of simpler operation, high sorting accuracy, and fast speed [21]. The advantage of the density gradient centrifugation method is that it is easy to operate, and the disadvantage is that it destroys the growth factors and the intact microenvironment of the original BMSCs, which is not conducive to BMSCs colonization. The most commonly used methods are flow cytometry and immunofluorescence staining, and changes in cell morphology can be observed using inverted microscopy as an aid to identification. Flow cytometry: There are mainly hematopoietic stem cells and BMSCs in the bone marrow, and BMSCs mainly express surface markers such as CD44 and CD90, but not CD34 and CD45, which are surface markers of hematopoietic cells. Immunofluorescence staining method: By identifying the surface antigen expression of BMSCs with immunofluorescence triple technique, bone marrow mesenchymal cells were observed to express CD29, CD90, and not CD45 under laser copolymer microscopy. Induction of in vitro directed differentiation of BMSCs into osteoblasts BMSCs in vitro osteogenic differentiation relies heavily on osteogenic induction medium, which includes Dex, sodium *β*-glycerophosphate (*β*-GP), and vitamin C (VitC), which are essential cofactors for the osteo-differentiation of BMSCs stem cells. Osteogenic capacity induces selective proliferation of BMSCs; stimulates the expression of core binding factor *α*1 (RUNX2), alkaline phosphatase (ALP), osteopontin (OPN) and osteocalcin (OCN); and increases the mRNA expression level of ALP. *β*-GP, as a source of phosphate in hydroxyapatite, provides phosphate ions, induces activation of ALP, and affects intracellular signaling molecules. VitC is a cofactor of collagen prolyl hydroxylase, regulates extracellular matrix collagen homeostasis, and enhances DNA activity to promote cell differentiation. In recent years, several different classes of substances have been reported to have the effect of promoting osteogenic differentiation of BMSCs in vitro, which can significantly improve the cellular purity of BMSCs [22]. Some herbal components have the effect of promoting osteogenic differentiation and proliferation of BMSCs, which is beneficial for the repair of bone defects. BMSCs were cultured in osteogenic induction medium containing Epimedium as the experimental group and without Epimedium as the control group. The results showed that the expression of osteogenic genes and the number of calcium nodules in the experimental group were significantly higher than those in the control group, confirming the synergistic effect of Epimedium and osteogenic induction medium in promoting osteogenic differentiation. The osteogenic induction medium of BMSCs was supplemented with different concentration gradients of osteopontin, and the results showed that osteopontin could promote osteogenic differentiation by regulating the expression of RUNX2 and OCN proteins, thus contributing to the maintenance of the dynamic balance of bone metabolism.

### 2.3. Deep Vision Methods

Medical image analysis initially focused on edge detection, texture features, morphological filtering, and the construction of shape models and template matching. These types of analysis methods are usually designed for specific tasks and are referred to as manual bespoke design methods. Machine learning analyzes the task in a data-driven manner and can automatically learn relevant model features and data characteristics from a large-scale dataset for a specific problem. Unlike models that are explicitly designed manually for a specific problem, machine learning methods automatically learn medical image features implicitly and directly from data samples, and the learning process is essentially an optimization problem-solving process. Through learning, the model selects the correct features from the training data, allowing the classifier to make the correct decisions when testing new data. Therefore, machine learning plays a crucial role in medical image analysis and has become the most promising area of research. Deep learning (DL) is a machine learning method that originated from the study of artificial neural networks and is motivated by the creation of neural networks that mimic the human brain to analyze and understand data. By observing how the visual center of the cat's brain processes retinotopic perceptual images, it was found that optic neurons process information in a hierarchical manner, with different neurons focusing on different object features, and each layer of neurons abstracting some of the object features for processing, with all information stimulated layer by layer, and the entire object perception stimulated at the highest layer of the center. The problem of gradient disappearance of BP algorithm is solved by adopting unlabeled datasets for network pretraining in deep feedforward networks. The unsupervised greedy layer-by-layer training method is used to effectively reduce the dimensionality of the observed objects, and then all network parameters are fine-tuned with supervised training. This algorithm brings hope for solving the deep structure-related optimization problem and has made a breakthrough in classification prediction such as image target recognition. Convolutional neural networks (CNNs), which use spatial relativity to reduce the number of parameters to improve training performance, were the first true multilayer structure learning algorithms. Long short-term memory (LSTM) has also made breakthroughs in image handwriting recognition and speech recognition. Deep learning has made important breakthroughs in several areas. In speech recognition, the introduction of Restricted Boltzmann machine (RBM) and Deep belief network (DBN) into speech recognition model training has been a great success in large vocabulary speech recognition systems, reducing the speech recognition error rate by 30% relative to the previous one. In its review, Harvard Medical School pointed out that the application of deep learning to solve medical image analysis tasks is the development trend in this field. In 2016, several experts have summarized, reviewed, and discussed the current state of research and problems of deep learning in medical image analysis and the reviews published in relevant journals have summarized the research on deep learning in medical image classification, detection and segmentation, and alignment and retrieval. The classical framework for CNN-based computer vision classification tasks is shown in Table 1.

## 3. Method

### 3.1. Model Architecture

Compared with traditional machine learning algorithms, visual deep learning algorithms avoid the tedious image preprocessing and feature extraction steps in traditional machine learning, and can be trained by directly inputting images, which can preserve more features and thus avoid errors and obtain higher recognition accuracy. In this paper, we use Convolutional Neural Network (CNN) as a feedforward network, whose neurons can locally connect adjacent neurons and preserve the spatial structure of the target through the special structure of the network, thus achieving a better performance in the field of image processing. For CNN, its input layer can be directly input to the original image, so it is widely used in many fields of computer vision, including image segmentation, image classification, and image understanding. In this paper, we directly input the obtained BMSCs maximum profile grayscale images into the designed CNN for model learning and training, and then use the obtained models for classification and recognition. The overall architecture of the proposed method is shown in Figure 4.

### 3.2. Method Details

For a normal Fully Connected Neural Network (FCN), it is basically the same as CNN in terms of structure with input and output and training process. Structurally, each node in CNN and FCN represents a neuron, and in FCN, all nodes in two adjacent layers are fully connected, while in CNN, nodes in two adjacent layers are locally connected. The input layer of CNN in image classification is the original picture of the image and the output layer represents the confidence level of different classification categories, which is consistent with the output of FCN. The biggest problem of using FCN images is that the fully connected layer has too many parameters, and they will cause the model to be computationally slow and prone to overfitting. The CNN consists of two types of structures, one is the feature extraction layer, where neurons are connected to the local receptive fields of the upper layer neurons and can be used to extract local features, and each local feature corresponds to a network structure. The other is the feature mapping layer, where each feature is considered as a plane with equal weights of the mapping neurons. The activation functions corresponding to the feature mapping structures are all displacement invariant. The convolutional layer in CNN is used for feature extraction, and this unique structure effectively reduces the feature resolution. Feature extraction process. At the same time, its structure has the feature of weight sharing, so parallel learning is possible. These two features make CNNs structurally closer to real biological neural systems, and they shine in the fields of natural language processing and image recognition. In addition, in practical applications, CNN can directly use the original image as input, learn features by using small input data, and retain the spatial relationship between the lower pixels, so that objects in the image can still be detected by the network when scene migration or image transformation occurs. Therefore, convolutional neural networks have the following advantages: they can learn with fewer parameters than fully connected neural networks; they can ignore the effects of classifying and recognizing the location of objects in the image and image distortion; and they can automatically learn and acquire features from the input data.

According to the role and function of each layer in CNN, they can be divided into the following five main types: input layer generally takes the vector form of a picture as input. Each layer input and output in FCN is a one-dimensional vector; and each layer input and output of CNN is arranged in three dimensions, similar to a rectangular body with three-dimensional dimensions of length, width, and depth. In computer graphics, the depth of the rectangle reflects the number of color channels in the image, which is 1 for grayscale images and 3 for RGB images. This part is called “filter” (Filter). The inner product of image and filter is the “convolution” operation, which is also the source of the name of convolutional neural network. In the computation process, data with certain dimensions (width ^*∗*^height ^*∗*^depth) are used as input and convolved with the filter to obtain a two-dimensional array. The process of filter forward propagation can be determined by setting the size of the filter and the depth of the node matrix is obtained by processing. Convolution kernel forward propagation is the process of getting the output of the next layer by the node output in the matrix of the previous layer through filter action. Suppose the height, width, and depth of the input region are *w*,*h*,*d*, respectively, and for the *i*-th node in the output unit node matrix, using bi to denote the corresponding bias in the *i*-th network node, the output value g(*i*) of the *i*-th node is

(1) $$\begin{array}{c} g\left(i\right)=f\left(\sum_{x=1}^{w}\sum_{y=1}^{h}\sum_{z=1}^{d}a_{x,y,z}\times w_{x,y,z}^{i}+b^{i}\right), \end{array}$$

where *x*,*y*, and *z* are the values of the filter node (*x*,*y*,*z*) and *f* is the activation function. The source pixel is obtained as the unit target pixel of the rightmost matrix by the inner product operation after the filter action.

When a picture (grayscale image) with depth (Depth) of only 1 is used as input, only the size of the filter needs to be set. The input can be converted into a one-dimensional vector expressing the tensor of the picture as the input of the network. The RGB color model is shown in Figure 5.  ^*∗*^h one-dimensional vector input, and the set of target pixels calculated by a filter is called the Feature Map, and the size of the area mapped on the original image by the pixel points on the feature map is called the Receptive Field. And, the common representation of the image is RGB color model with 3 channels. The following equation indicates the size and parameters of the filter, and *r*, g, and *b* in the lower corner indicate the weights of the red (red), green (green), and blue (blue) color channels, respectively.

(2) $$\begin{array}{c} \left[\begin{array}{cc} w_{r1} & w_{r2}\\ w_{r3} & w_{r4} \end{array}\right],\left[\begin{array}{cc} w_{g1} & w_{g2}\\ w_{g3} & w_{g4} \end{array}\right],\left[\begin{array}{cc} w_{b1} & w_{b2}\\ w_{b3} & w_{b4} \end{array}\right]. \end{array}$$

The filters then move up the input image in a certain order from the top left corner to the bottom right corner, and the distance of each move is called the stride. The relationship between the size of the input matrix (input_size), the size of the filter (filter_size), and the size of the output matrix (output_size) is satisfied as follows:

(3) $$\begin{array}{c} \text{output}\_\text{size }=\frac{\text{ output}\_\text{size}-\text{filter}\_\text{size }}{\text{ stride }}+1. \end{array}$$

### 3.3. Data Enhancement

For the classification recognition model of convolutional neural networks, there is a conclusion that

(4) $$\begin{array}{c} P\left(\text{ test error}\leq \text{training error }+\sqrt{\frac{h\left(\text{log}\left(2N/h\right)-\text{log}\left(\left(\eta /4\right)\right.\right)}{N}}\right)=1-\eta . \end{array}$$

In the above equation, N is the number of training samples and *h* is the VC dimension of the classification model, where the root part is the model complexity penalty term. If the training model can make the training error rate very low and the model complexity penalty term very low, the test error rate can be guaranteed to be at a very low level. For the model complexity penalty, the smaller the *h*, the smaller the penalty, and the larger the N, the smaller the penalty. Deep learning models often have a large VC dimension and need a larger number of training samples to reduce the penalty term; therefore, deep network structures like CNNs need large samples for model training to avoid overfitting. Due to the high cost of obtaining confocal microscopic images of BMSCs, the difficulty of related biological experiments, and the limited number of images with labels judged by combining protein expression determination and doctors' clinical experience, a total of 128 samples are available, and data augmentation is needed for the BMSCs dataset.

## 4. Experimentation and Evaluation

### 4.1. Dataset

In order to prevent the model from overfitting, data augmentation is needed for the obtained 128 example samples. The ImageDataGenerator() module in keras can implement the basic data augmentation function. This function can be used to generate augmented data cyclically during training until the iteration is completed. The function has several operations that can be used to augment the image data with different assignments. Seven data augmentation functions are selected, such as rotation, flip, translation, scale transformation, noise perturbation, color dithering, and contrast. The 128 samples are augmented to 1200, and 900 are selected as training samples and 300 as test samples. The maximum profile image of BMSCs is obtained as the input, and its resolution is 1000 × 1000. In order to reduce the model computation and improve the computing efficiency, Gaussian Pyramid algorithm is used to downsample the image, so that its resolution is reduced to 64 × 64. This set of images obtained is used as the input of BMSCs classification recognition network. The GoogleNet (InceptionV3) model is borrowed and fine-tuned using Fine-Tune to obtain the recognition accuracy of the model for BMSCs.

### 4.2. Experimental Steps

The experimental hardware platform uses Inteli7-7700k processor, DDR4-16G memory, and GeForce1060 graphics card (CUDA acceleration module is available). The implementation of InceptionV3 classification and recognition algorithm is mainly based on the Keras library of *Python* platform, and the model is trained using Fine-Tuning, and then the main process is as follows: 1. Define the function and load the module. Import the InceptionV3 model and load the corresponding function modules. 2. Set the size of the imported images, the number of nodes in the fully connected layer, and the number of frozen layers; set the training set and validation set parameters and then use ImageDataGenerator() for data augmentation and image generation. 3. Fine-tuning (Fine-Tuning). After adding a new layer with the set number of classifications and base model, all previous layers are frozen and the correct bottleneck features are obtained to train the network layer by layer. 4. Classification and recognition. Load the trained new model and perform classification and recognition for the test set images. Among them, blue is the rising curve of the accuracy of the training set and green is the rising curve of the accuracy of the test set. Finally, after 10,000 iterations, the accuracy of the test set is 0.989, which achieves an excellent classification and recognition effect.

### 4.3. Comparison of Results

Table 2 shows the comparison of the classification recognition rates and time consumption of the three classification recognition models for BMSCs, showing that the convolutional neural network has a higher accuracy rate for the classification recognition of images and achieves the expected results of the experiments.

### 4.4. Ablation Experiments

According to the experimental results, the accuracy of classification recognition of BMSCs varies with the same batch size, learning rate, activation function, and number of iterations due to the different structure of the network, which proves that the deeper layers of the network have some advantages in the accuracy of recognition. The MLP with 3 implied layers and 3,5,3 neurons per layer achieves the same highest classification rate as the MLP with 4 implied layers and 3,3,5,5 neurons per layer, but due to its simpler model with fewer training parameters, it is selected as the final MLP structure for the classification of BMSCs. The accuracy of different network structures of MLP in identifying normal and senescent cells in BMSCs is shown in Table 3.

## 5. Conclusion

The incidence of intracanalicular deformity and osteochondral deformity differs significantly between types, and those with combined osteochondral deformity are more likely to have intracanalicular deformity. Bone marrow mesenchymal stem cells have a wide range of clinical applications as stem cells that play an important role in supporting the proliferation of hematopoietic and hematopoietic progenitor cells, regulating the bone marrow microenvironment, and have the potential for multi-directional differentiation. Morphology-based taxonomic identification is of great significance for the evaluation of their physiological functions. In this paper, based on the optical sections of fluorescence confocal laser microscope, morphological features were extracted, and various models were designed on the *Python* platform using machine learning methods for algorithm development and validation. The main contents include the preprocessing of optical sections, the calculation of the maximum profile of the cell 3D structure, the calculation and selection of cell features, and the design and implementation of machine learning models. In this paper, based on the selected cell features, we propose an algorithm based on visual depth, use the data augmentation method to realize the expansion of small sample cell data, and use the migration learning method to build a network structure suitable for the classification and recognition of this topic by InceptionV3 through the Fine-Tuning method to realize the classification and recognition, and the recognition accuracy is improved compared with the traditional machine learning method by up to 98.9%. However, this algorithm learns a specific set of expressions for a specific task, rather than learning a general model that can be fully migrated. Therefore, in the future, we need to study the generalization performance of the model to make the model have strong adaptability, so that it can be widely used in a variety of diseases.

## Figures and Tables

**Figure 1:** Schematic diagram of the genes involved in the typing of vertebral defects.

**Figure 2:** Cell morphology of BMSCs under transmission electron microscopy.

**Figure 3:** Morphology of primary and passaged bone marrow mesenchymal stem cells.

**Figure 4:** Model structure.

**Figure 5:** RGB color model schematic.

**Table 1:** CNN-based classical framework for computer vision classification tasks.

Network structure	Features	Remarks
LeNet	Multiple convolutional layers and subsampling layers	American handwritten digit recognition
AlexNet	ReLU and dropout are proposed	Set a new world record in the ImageNet ILSVRC 2012 object classification competition
VGGNet	Proposed to use small convolution to verify deeper networks and multi-scale fusion	Winner of ILSVRC 2014 for localization task and runner-up for classification task
GoogleNet	22-Layer network with multiple inception structures in series	Winner of ILSVRC 2014 classification and detection task
ResNet	Proposed residual net, introduced jump connection, 152 layers deep	Winner of the ILSVRC 2015 object detection and object recognition competition
Inception ResNet	Inception structure combined with residual net	Achieves comparable performance to ResNet, but with faster convergence
FCN	Densities prediction for pixel-level classification	Avoids duplicate convolution computation due to overlap between image blocks
DenseNet	Direct connection between any two layers	Mitigates gradient disappearance, enhances feature propagation, supports feature reuse, and reduces the number of network parameters
SqueezeNet	Simplify network structure and reduce network parameters	Achieve the same accuracy of AlexNet with only 1/50th of the number of AlexlNet parameters
DCNN	Proposed deformable deep convolutional neural network	Enhances the network's ability to model geometric transformations
DPN	Combines the advantages of ResNet and DenseNet	The DPN-based team won the 2017 ILSVRC object detection and object recognition competition
SENet	Learn the importance of each feature channel and reinforce useful features	Winner of the 2017 ILSVRC image classification task competition

**Table 2:** Comparison of the recognition accuracy and time consumption of normal and aging BMSCs by different machine learning models.

Model	Svm	MLP	Inception V3
Average recognition rate	0.978	0.960	0.989
Time consuming	2.935s	1.762s	0.531s

**Table 3:** Accuracy of normal versus senescent cell recognition in BMSCs with different network structure MLPs.

Network structure	3 ^*∗*^3	5 ^*∗*^3	3 ^*∗*^5	3 ^*∗*^3 ^*∗*^3	3 ^*∗*^5 ^*∗*^3	3 ^*∗*^3 ^*∗*^5	3 ^*∗*^3 ^*∗*^5 ^*∗*^5
Group 1	0.868	0.868	0.868	0.921	1.000	0.921	0.973
Group 2	0.842	0.895	0.868	0.973	0.921	1.000	0.947
Group 3	0.868	0.921	0.921	0.947	0.921	0.921	0.921
Group 4	0.895	0.895	0.921	0.973	1.000	1.000	1.000
Group 5	0.842	0.842	0.895	0.921	0.947	0.947	0.947
Group 6	0.895	0.921	0.895	1.000	0.973	0.947	0.973
Average recognition rate	0.868	0.890	0.895	0.956	0.960	0.956	0.960

## Data Availability

The datasets used during the current study are available from the corresponding author on reasonable request.
